The article "Analysis of the Correlation of Basic Fibroblast Growth Factor in Serum of Patients with Diffuse Large B-Cell Lymphoma with Clinicopathological Efficacy and International Prognostic Index" was retracted in 2023. Reasons: signs of a paper mill; suspected computer-generated content; unreliable results or conclusions; lack of ethics approval or compliance.

# Analysis of the Correlation of Basic Fibroblast Growth Factor in Serum of Patients with Diffuse Large B-Cell Lymphoma with Clinicopathological Efficacy and International Prognostic Index

**DOI:** 10.1155/2022/8311535

**Published:** 2022-09-19

**Authors:** Yan Pan, Pinjiang Han, Fengmei Fang, Haijuan Xiao, Lijing Zhu, Juan Pu, Panfei Hou

**Affiliations:** ^1^Department of Clinical Laboratory, Lianshui People's Hospital Affiliated to Kangda College of Nanjing Medical University, Huai'an 223400, China; ^2^Department of Radiotherapy, Lianshui People's Hospital Affiliated to Kangda College of Nanjing Medical University, Huai'an 223400, China

## Abstract

The correlation of basic fibroblast growth factor (bFGF) in serum of patients with diffuse large B-cell lymphoma (DLBCL) with clinicopathological efficacy and International Prognostic Index (IPI) is analyzed. 115 DLBCL patients admitted to our hospital for treatment from June 2020 to June 2021 are selected as the DLBCL patient group, 65 healthy subjects who received physical examination in our hospital during the same period are selected as the healthy control group, and the serum bFGF levels of DLBCL group and healthy control group are observed before treatment. The experimental results show that the serum bFGF expression of DLBCL patients is decreased significantly after chemotherapy, and the serum bFGF expression of DLBCL patients is closely related to the treatment effect, disease progression, tumor invasion, and prognosis, which has important clinical significance for judging the disease, treatment effect, and prognosis of patients.

## 1. Introduction

Diffuse large B-cell lymphoma (DLBCL) is a common type of non-Hodgkin's lymphoma, accounting for about 30%∼40% of all lymphomas, with highly invasive and rapidly progressive characteristics [1]. Active evaluation of tumor progression, treatment effect, and prognosis of patients can provide an important reference for clinical treatment intervention [2, 3]. Previous studies have pointed out that serum bFGF detection in DLBCL patients can help clinicians better evaluate the patient's condition, clarify clinical analysis, predict prognosis, and then optimize and improve clinical diagnosis and treatment plans [4]. It should be noted that although the single serum bFGF index detection model has been applied to evaluate the disease progression and prognosis of DLBCL patients, there are still some limitations and deviations [5]. Above all, in order to further optimize and improve the clinical detection mode, 115 DLBCL patients and 65 healthy subjects are selected for detection and analysis in this study, and the correlation between serum bFGF and IPI score is observed, in order to further explore the mechanism of serum bFGF influencing the disease development and prognosis.

The rest of this paper is organized as follows: Section 2 discusses related work, followed by clinical information and the proposed treatment method designed in Section 3.  Section 4 shows the experimental results and analysis, and Section 5 briefly summarizes all of the standpoints of the whole text.

## 2. Relate Work

DLBCL is a common clinical invasive tumor with complex clinical manifestations, which endangers people's health [6]. Tumor metastasis and invasion are the biggest cause of tumor treatment and the main cause of death in patients. The invasion, growth, metastasis, and prognosis of solid tumors are closely related to angiogenesis and become a new standard for monitoring tumor development [7]. One of the most important regulatory factors of neovascularization is bFGF [8]. With the development of medical science and technology, the application of protein detection in disease judgment and diagnosis is promoted. The detection of serum bFGF factor levels has become the standard for tumor detection [9]. Studies have shown that invasion and metastasis are significantly related to the high expression of bFGF in solid tumors such as colorectal cancer and liver cancer [10]. Clinically, because DLBCL has no clear diagnostic and prognostic indicators, in order to accurately reflect the condition of such patients, the level of serum bFGF factor is used to judge the diagnosis and prognosis of DLBCL [11].

In this study, the serum bFGF levels of DLBCL patients and healthy subjects were detected and analyzed. The results showed that the serum bFGF levels of DLBCL patients before treatment were significantly higher than that of healthy subjects. In order to further verify the influence of serum bFGF expression on the degree of disease in DLBCL patients, this study compared serum bFGF expression in DLBCL patients with different clinical stages and showed that with the increase in the clinical analysis of patients, serum bFGF also showed a high expression trend. Previous literature have pointed out that IPI scores can reflect the treatment response, recurrence, and survival of lymphoma patients to a certain extent [12]. The results of this study showed that there was a positive correlation between serum bFGF level and IPI score in DLBCL patients, which suggested that there was a close relationship between serum bFGF level and the condition of DLBCL patients. After 1 course of treatment, the level of serum bFGF in DLBCL patients decreased significantly, and the higher the clinical stage, the greater the reduction. The reason may be in the process of angiogenesis, the bFGF can use the endothelial cells of patients with DLBCL efficient tyrosinase receptors in vascular endothelial cells to induce the proliferation, and promote blood vessel formation. The generation of vascular permeability is higher, easy to penetrate plasma proteins to the extracellular matrix, which is more conducive to the growth of fibroblasts and endothelial cells, Vascular rich tumor matrix is formed to promote tumor invasion and metastasis [13]. With the increase in the clinical stage, tumor blood vessels in DLBCL patients are gradually enriched, which is more conducive to tumor cell infiltration and growth, and the expression of bFGF in patients increases accordingly [14]. It also indicates that the CHOP regimen can inhibit tumor cell growth and destroy the tumor growth environment in DLBCL patients to a certain extent, which can result in reduced neovascularization and reduced serum bFGF level.

The bFGF, a member of the FGFs family, is a kind of polypeptide growth factor widely existing in the body. It exists in tumor tissues and binds to its receptors and has a wide range of physiological, pathological, and biological activities in various tissues of the body. Studies have shown that bFGF can promote the angiogenesis of solid tumors, which is an indirect indicator of tumor angiogenesis and is closely related to tumor growth, invasion, metastasis, and prognosis [15]. The formation of blood vessels to diffuse large B-cell lymphoma in growth, progression, and metastasis is very important. The bFGF is in the process of the formation of diffuse large B-cell lymphoma vascular specificity is high; it can effect on vascular proliferation factor, make use of tyrosinase in endothelial cells receptors on endothelial cells effectively, induce endothelial cell proliferation, and thus, promote the formation of blood vessels. Meanwhile, the new blood vessels induced by bFGF have high permeability, and the plasma proteins in the circulation process are easy to penetrate into the extracellular matrix, which can provide a good growth environment for endothelial cells and fibroblasts to form a tumor matrix rich in blood vessels; thus, provide conditions for tumor metastasis and invasion [16]. As vascular regenerative factors, bFGF and its receptor have been recognized as key factors in the generation of mediated angiogenesis. It can act on vascular endothelial mitosis and form new blood vessels and is the strongest cytokine to promote tumor angiogenesis [17].

## 3. Clinical Information and the Proposed Treatment Method

### 3.1. Clinical Information

A total of 115 DLBCL patients admitted to our hospital for treatment from June 2020 to June 2021 are included in the DLBCL patient group, and 65 healthy subjects who received physical examination in our hospital during the same period are selected as a healthy control group. In the DLBCL patient group, there are 61 males and 54 females, aged from 45 to 75 years old, with an average of (56.32 ± 4.58) years old. Body mass index (BMI) ranged from 18.14 to 26.47 kg/m^2^, with an average of (24.16 ± 2.05) kg/m^2^. Clinical stages: There are 21 stage I patients, 25 stage II patients, 30 stage III patients, and 39 stage IV patients. In the healthy control group, there are 37 males and 28 females, aged from 42 to 73 years old, with an average of (55.74 ± 4.36) years old. BMI ranged from 18.22 to 26.58 kg/m^2^, with an average of (23.87 ± 1.94) kg/m^2^. There are four inclusion criteria for DLBCL patients (1) all patients who received treatment for the first time are >18 years old; (2) all patients underwent biopsy or clinicopathological examination, and their clinical manifestations and diagnostic results are consistent with WHO classification of malignant lymphoma [18]; (3) the clinicopathological data of the patients are complete; (4) patients with high clinical compliance can cooperate to participate in this study and related investigations until the end of the study.

### 3.2. The Proposed Treatment Method

#### 3.2.1. Chemotherapy Regimen

All DLBCL patients receive CHOP chemotherapy. On the first day of chemotherapy, intravenous infusion of cyclophosphamide (Harbin Sanlian Pharmaceutical Co., LTD., National Drug Approval LETTER H20084195) (dosage set as 750 mg/m^2^), adriamycin (Shanxi Pude Pharmaceutical Co., LTD., National drug Approval H14023143) intravenous infusion (dose set at 50 mg/m^2^), vincristine (produced by Zhejiang Haizun Pharmaceutical Co., LTD., National drug approval H20043326) intravenous infusion (dose set at 1.4 mg/m^2^); five days before chemotherapy, prednisone (Shanxi Sun Simimiao High-tech Pharmaceutical Co., LTD., National Drug approval H61020333) intervention therapy is taken orally at 100 mg/d, and the above medication regimen is one course of treatment, and then the next course of treatment is continued after 16 days of drug withdrawal.

#### 3.2.2. Detection Method of Serum bFGF

8 mL fasting venous blood is taken from the DLBCL group before chemotherapy intervention and in the morning after one course of chemotherapy intervention, and 8 mL fasting venous blood is taken from healthy subjects in the healthy control group on the day of physical examination. A centrifuge is used to complete centrifugation with parameters set at 3500 r/min, centrifugation radius of 10 cm, and duration of 10 min. Then the supernatant is taken and the serum bFGF levels of the two groups are detected by double-antibody sandwich ELISA. The kit is purchased from Shanghai Seeger Biotechnology Co., LTD., and all related operations during the test are strictly carried out according to the kit instructions.

### 3.3. Observation Indicators

There are four observation indicators as follows: (1) the serum bFGF levels of the DLBCL group and healthy control group are compared before treatment; (2) the serum bFGF levels of patients with different stages of DLBCL are compared before and after treatment; (3) the serum bFGF levels and IPI scores of patients with different prognosis are compared; (4) the correlation between serum bFGF expression and prognosis of DLBCL is analyzed.

### 3.4. International Prognostic Index (IPI) Scoring Criteria

After 1 course of treatment, complete disappearance or reduction of lesions ≥ 50% is considered as improvement. The lesions are reduced by less than 50% or even increased to worsen. IPI scores are performed on DLBCL patients before and after 1 course of treatment. Patients with age > 60 years old, clinical stage III or IV, systemic status score ≥ 2 points, ≥ 2 extranodal lesions, and elevated serum lactate dehydrogenase level are counted as 1 point, and the total score is 0–5 points. The higher the IPI score, the higher the severity of the patient's disease [19].

### 3.5. Statistical Methods

SPSS 26.0 software is used for statistical analysis of the data generated in this study. The measurement data are expressed as mean ± standard deviation ($\bar{x}$ ± *s*) after normal distribution, and the comparison is completed by the *t/F* test. Pearson correlation coefficient is used to analyze the correlation between serum bFGF expression and the prognosis of DLBCL patients.

## 4. Experimental Results and Analysis

### 4.1. Comparison of Serum bFGF Levels before Treatment

Table 1 shows the comparison of serum bFGF levels between the DLBCL group and the healthy control group before treatment. It can be seen from Table 1 that serum bFGF expression in the DLBCL group is increased significantly more than that in the healthy control group (*P* < 0.05) before treatment.

### 4.2. Comparison of Serum bFGF Levels in Patients with Different Stages of DLBCL

Subgroups are established according to the clinical stages of DLBCL patients admitted to our hospital, including stage I DLBCL patients group, stage II DLBCL patients group, stage III DLBCL patients group, and stage IV DLBCL patients group.  Table 2 shows the serum bFGF levels in patients with different clinical stages of DLBCL. In Table 2, ∗ is compared with before treatment, *P* < 0.05; ^a^ is compared with the group of stage I DLBCL group, *P* < 0.05; ^b^ is compared with the group of stage II DLBCL patients, *P* < 0.05; ^c^ is compared with the group of stage III DLBCL patients, *P* < 0.05. It can be seen from Table 2 that the serum bFGF levels in all groups are significantly different and increased with the increase in the clinical stage before the treatment. After the treatment, serum bFGF levels in all groups decreased significantly from those before the treatment, and there are statistically significant differences (all *P* < 0.05).

### 4.3. Comparison of the Serum bFGF Levels and IPI Scores of Patients with Different Prognosis

The prognosis of DLBCL patients is observed after one course of treatment and a subgroup is established. Patients who improved after treatment are included in the improved GROUP of DLBCL patients (*n* = 73) and patients who deteriorated after treatment are included in the deteriorated group of DLBCL patients (*n* = 42).  Table 3 shows the comparison of serum bFGF levels and IPI scores in patients with different prognoses. In Table 3, *∗* represents a comparison with before treatment, *P* < 0.05. It is clearly evident from Table 3 that the serum bFGF level and IPI score of patients in both groups decreased significantly than before after treatment, and the serum bFGF level and IPI score of patients in the DLBCL improvement group decreased significantly than the DLBCL deterioration group (all *P* < 0.05).

### 4.4. Analysis of the Correlation between Serum bFGF Expression and Prognosis of DLBCL Patients

Figure 1 shows the correlation between serum bFGF expression and IPI score. It can be seen from Figure 1 that there is a significant positive correlation between bFGF expression and IPI score in DLBCL patients (*P* < 0.05).

## 5. Conclusion

The correlation of bFGF in the serum of patients with DLBCL with clinicopathological efficacy and IPI is analyzed. The level of serum bFGF in DLBCL patients can reflect the patient's condition, predict the patient's pathological stage and judge the prognosis, which has a certain clinical guiding value.

## Figures and Tables

**Figure 1:** Correlation between serum bFGF expression and IPI score.

**Table 1:** Comparison of serum bFGF levels between the DLBCL group and the healthy control group before treatment (ng/mL, $\bar{x}$ ± *s*).

Group	The number of cases	Serum bFGF
A group of patients with DLBCL	115	26.17 ± 2.86
Healthy control group	65	17.25 ± 1.72
*t*	—	20.897
*P*	—	＜0.001

**Table 2:** Serum bFGF levels in patients with different clinical stages of DLBCL (ng/mL, $\bar{x}$ ± *s*).

Group	Before the treatment	After the treatment
Stage I DLBCL patients group (*n* = 21)	19.36 ± 2.04	15.17 ± 1.15^*∗*^
Stage II DLBCL patients group (*n* = 25)	22.13 ± 2.11^a^	18.95 ± 1.52^*∗*^^a^
Stage III DLBCL patients group (*n* = 30)	27.04 ± 2.32^ab^	20.27 ± 1.61^*∗*^^ab^
Stage IV DLBCL patients group (*n* = 39)	33.18 ± 2.46^abc^	24.47 ± 1.79^*∗*^^abc^
*F*	8.176	7.549
*P*	＜0.001	＜0.001

**Table 3:** Comparison of serum bFGF levels and IPI scores in patients with different prognoses ($\bar{x}$ ± *s*).

Group	Serum bFGF (ng/mL)		IPI score (score)	
	Before the treatment	After the treatment	Before the treatment	After the treatment
DLBCL patients improved group (*n* = 73)	21.07 ± 1.62	16.12 ± 1.59^*∗*^	3.48 ± 0.51	1.81 ± 0.24^*∗*^
DLBCL patients deteriorated group (*n* = 42)	25.68 ± 2.25	21.74 ± 2.18^*∗*^	3.97 ± 0.55	2.86 ± 0.36^*∗*^
*T*	−12.707	−15.890	−4.820	−18.737
*P*	＜0.001	＜0.001	＜0.001	＜0.001

## Data Availability

The simulation experiment data used to support the findings of this study are available from the corresponding author upon request.
